# Laser CO_2_ treatment for vulvar lymphedema secondary to gynecological cancer therapy: A report of two cases and review of the literature

**DOI:** 10.3892/ol.2015.2961

**Published:** 2015-02-12

**Authors:** FRANCESCO SOPRACORDEVOLE, FRANCESCA MANCIOLI, VINCENZO CANZONIERI, MONICA BUTTIGNOL, GIORGIO GIORDA, ANDREA CIAVATTINI

**Affiliations:** 1 Department of Gynecological Oncology, Oncological Referral Center, National Cancer Institute, Aviano, Pordenone 33081, Italy; 2 Department of Woman’s Health Sciences, Polytechnic University of Marche, Ancona 60123, Italy; 3 Division of Pathology, Oncological Referral Center, National Cancer Institute, Aviano, Pordenone 33081, Italy

**Keywords:** vulvar lymphedema, lymphorrhea, pelvic radiotherapy, pelvic lymphadenectomy

## Abstract

Vulvar lymphedema is an uncommon and disabling side-effect of pelvic lymphadenectomy and pelvic radiotherapeutic treatment for invasive genital cancer. Lymphorrhea, a complication of lymphedema, may be extremely distressing for patients due to the requirement to wear sanitary towels and as the pain and loss of elasticity of the vulvar skin and mucosa can cause discomfort during coitus. Surgical treatments of lymphorrhea and vulvar lymphedema secondary to gynecological cancer treatments remain controversial and are not currently considered to be the standard therapy. The present study reports two cases of vulvar lymphedema complicated by vulvar lymphorrhea in females who had undergone treatment for cervical and endometrial cancer, respectively; a review of the literature is also included. In the two present cases, vulvar lymphedemas were refractory to standard treatments, including decongestive therapy, manual lymph drainage, elastic bandaging, low-stretch bandaging, exercises and skin care. Laser CO_2_ excision and vaporization of the whole skin and mucosal tissue of the vulva was successfully performed to treat the lymphorrhea and improve quality of life. Thus, the present two cases indicated that laser CO_2_ surgery may present an additional therapy for the treatment of genital lymphedema that is refractory to other treatments.

## Introduction

Lymphedema is the chronic and progressive engorgement of tissues caused by deficient lymphatic drainage (1). Vulvar lymphedema is one of the most disabling side-effects of treatment for gynecological cancers involving systematic pelvic, or pelvic and aortic, lymph node dissection associated with adjuvant or neoadjuvant radiation therapy (1). Lymphorrhea may occur as a complication of lymphedema (1,2). The incidence of genital lymphedema is unknown, as it is frequently undiagnosed (2). As with other types of lymphedema, the condition typically occurs in the first three to four years after cancer treatment, however, it may develop up to 30 years later (1). Genital lymphedema is typically combined with lower limb lymphedema; systematic pelvic lymph node dissection damages the lower limb lymphatic system, leading to a reduced capacity to absorb excess water and cells from the interstitial space (2). Treatment using compressive pump (or bandaging) therapy may subsequently lead to an increase in vulvar lymphatic load, followed by the appearance of dilated lymphatic vessels and vulvar lymphedema. In addition to skin alterations, a significant symptom is lymphorrhea, which occurs following increases in tissue pressure, causing fluid to leak from the thin layer of skin. Furthermore, edematous skin is an ideal medium for bacteria and can lead to a high risk of developing skin infections, particularly erysipelas (3). Lymphorrhea may be extremely distressing for patients due to the requirement to wear sanitary towels, and as the pain and loss of elasticity of the vulvar skin and mucosa can make coitus uncomfortable, with altered vulvar/vaginal sensation (4).

Few previous studies have been published with regard to the management of vulvar lymphorrhea and lymphedema secondary to radical treatment for gynecological cancer. The current study reports two cases involving the development of late symptoms of vulvar lymphedema in females who had previously undergone treatment for gynecological cancers. The condition was refractory to standard therapies in these cases and thus, laser CO_2_ surgery was performed. Laser CO_2_ surgery is a technique used for the excisional conservative treatment of preinvasive and initially invasive neoplasia of the lower female genital tract (5). In the current study, this surgical technique acted to induce a coagulative sclerosis in order to obliterate the subcutaneous and submucosal lymphatic channels, and create a fibrous layer capable of preventing the lymphorrhea. Written informed consent was obtained from both patients.

## Case report

### Case one

In 1986, a 29-year-old female underwent a Piver type III radical hysterectomy, systematic pelvic lymphadenectomy, adjuvant pelvic radiotherapy (50.60 Gy) and vaginal brachitherapy (20.34 Gy) for the treatment of International Federation of Gynecology and Obstetrics (FIGO) stage IB1 pN1 cervical cancer (6). At six months post-treatment, bilateral lower-limb lymphedema developed. Lymph drainage and elastic bandaging were performed with limited efficacy. In 1988, the patient experienced difficulties due to chronic lower-limb lymphedema.

In 2003, a painful vulvar edema developed, followed by vulvar lymphorrhea. In 2004, the patient was referred to the Department of Gynecological Oncology of the Aviano National Cancer Institute (Pordenone, Italy), due to a worsening in vulvar pain, classified as a score of 9 according to the Visual Analog Scale (VAS) for pain evaluation (7). The patient reported a dragging, heavy and bursting sensation, resulting in the loss of sexual function and difficulties in urination, with no evidence of urinary infection.

A vulvar examination revealed swollen inner and outer labia and vulvar edema, with associated fibrosis and skin changes, including thickening, dryness and hyperkeratosis. A vulvar specimen measuring 2.0×0.7×0.2 cm was excised, and a clinical diagnosis of vulvar lymphedema was confirmed by histological examination of the lesion, which revealed acanthosis, multiple dilated lymph vessels lined by a single layer of endothelium in the upper dermis, downward growth of the epidermis, a lymphoplasmacytic inflammatory infiltrate and an absence of giant or atypical cells (Fig. 1). Computed tomography and ultrasound scans of the abdomen were conducted, revealing no evidence of associated lymphoceles or recurrence of pelvic or retroperitoneal disease.

Vulvar excisional and vaporization treatment was performed in four sessions using a colposcopy-guided CO_2_ laser, with a constant emission power of 20 W/cm^2^ and a beam diameter of <0.2 and 0.5–1 mm for resection and vaporization, respectively, under local anesthesia with 2% mepivacaine. Excisional treatment was performed to obtain additional specimens in order to further investigate potential concurrent causes of vulvar edema. The depth of excision/vaporization was 0.3 cm, up to the sub-epithelial tissue. The procedures were performed as day surgery without antibiotic prophylaxis, and no complications occurred. Following recovery from the treatment, the patient experienced relief from the aforementioned pain and heaviness, subsequent to the resolution of the lymphorrhea. A pain assessment was performed every six months during follow-up gynecological examinations, with VAS scores (7) ranging from 0–2. A vulvar biopsy performed six months after vaporization treatment revealed multiple dilated lymph vessels without edema. The patient experienced a recurrence of vulvar lymphorrhea seven years after the treatment, which was again treated by laser CO_2_ vaporization, as previously described, resulting in a reduction of the persistent symptoms.

### Case two

In 1997, a 49-year-old female underwent a Piver type III radical hysterectomy with systematic pelvic lymphadenectomy and adjuvant pelvic radiotherapy (45 Gy) for the treatment of FIGO stage II, pN0, G3 endometrial adenocarcinoma (6).

Beginning in 2002, the patient suffered with recurrent vulvar erysipelas and chronic vulvar edema, secondary to lower-limb lymphedema, which was partially treated by combined decongestive therapy consisting of compressive bandaging and manual lymph drainage.

In 2012, the patient was referred to the Department of Gynecological Oncology of Aviano National Cancer Institute due to gradually increasing swelling of the vulva over a period of six months, associated with a genital pain score of 4–5 according to a VAS evaluation (7); the symptoms prohibited regular physical and sexual activity. A gynecological examination revealed multiple, firm, hyperkeratotic glossy papules and swelling of the vulva associated with changes in skin texture and leakage of serous fluid through the skin (lymphorrhea). A vulvar biopsy measuring 1.0×0.8×0.3 cm was used to determine a diagnosis of vulvar lymphedema (Fig. 2). As the standard treatments for lower-limb lymphedema were ineffective in improving the vulvar symptoms, vulvar excisional and vaporization treatments (three sessions) were performed using colposcopy-guided laser CO_2_ (as described in case one). Due to the patient’s history of erysipelas, a three-day regimen of the antibiotic azithromycin (500 mg/day) was administered. No complications were experienced, and the symptoms of pain and heaviness were relieved following reduction of the edema. During the 24-month follow-up examination, the patient presented with mild vulvar lymphedema without symptoms (VAS score, 0) and without lymphorrhea.

A biopsy performed in 2013 revealed a reduction in the dilatation of the dermal vessels, associated with moderate fibrosis (Fig. 3).

## Discussion

Lymphedema is a chronic and frequently incurable condition that may occur following therapeutic interventions affecting lymphatic drainage mechanisms, such as the surgical treatment of cancer (8). Histological examination may be used to determine the diagnosis of lymphedema, which is characterized by dilated and tortuous lymphatic vessels lined by a single layer of flat endothelial cells. Secondary changes (primarily atrophic) are typically observable in the overlying epidermis, in addition to inflammatory infiltrates, with slight fibrosis of the dermis. A number of histological features of vulvar lymphedema may mimic aggressive angiomyxoma; therefore this differential diagnosis must be considered, along with other myxedematous tumors of the vulvovaginal region (9). Vulvar lymphedema is typically secondary to lower limb lymphedema, following lymphadenectomy for the treatment of gynecological cancer (2). Although lower limb lymphedema has been extensively investigated, few studies are available with regard to vulvar lymphedema. Lymphedema of the female external genitalia following lymphadenectomy may be initially asymptomatic, or characterized by minimal symptoms that are often not reported by the patient. Later, the condition may severely impair the quality of life of affected patients, inducing aesthetic alteration and, particularly when associated with lymphorrhea, causing discomfort and pain during walking, sexual activity or when lying down, as well as recurrent erysipelas (3,4).

Lymphatic physiopathology is poorly understood; it has been hypothesized that the combination of surgery and adjuvant treatment may lead to fibrosis, with a subsequent obliteration of the lymphatic vessels and failure of lymph drainage, resulting in chronic and progressive tissue engorgement (10). This condition is exacerbated by lower-limb lymphedema as a consequence of a prior defect in lymph drainage. The proper management of lymphedema involves patient education to detect symptoms that are indicative of early disease onset, including heaviness, skin tightness, aching, numbness, weakness, impaired limb function or pain; no definitive effective therapy has been determined, and there are few studies available with regard to the treatment of female genital lymphedema and vulvar lymphorrhea (1).

A number of surgical approaches for the treatment of limb lymphedema refractory to conservative decongestive methods have been proposed. Lymphaticovenular anastomosis using an autologous interposition vein graft has been reported to be effective, simple to perform and minimally invasive for the treatment of secondary lymphedema of the upper and lower extremities (11). This supermicrosurgery technique facilitates bypassing the region of lymph flow obstruction, providing an alternative route for lymphatic fluid recirculation into the venous system through multiple lymphatic-venous or lymphatic-venous-lymphatic anastomoses (11,12).

Autologous or heterologous transplantation of vascularized lymph nodes has also been proposed (11); this tissue may prevent retroperitoneal fibrosis following lymphadenectomy, and allows neuromatous structure reconstitution, with pain relief. The nodes appear to survive well, and establish connections with locally situated lymph vessels, which assists in lymphatic return if the vasculature is microsurgically connected (13). Microsurgery and reconstructive surgery have also been proposed to treat lymphedema of the external male genitalia, a frequent complication of pelvic radical surgery following pelvic lymphadenectomy (14,15).

Lymphangiography has been demonstrated to be a valuable tool in the treatment of lymphedema, and acts to induce an inflammatory reaction that closes the leak (16). One previous study reported three cases of groin nodal ultrasound-guided lymphangiography for the diagnosis and treatment of genital lymphedema (16). Transnodal Lipiodol injection facilitates the visualization of nodal and lymphatic vessels. It has been hypothesized that Lipiodol accumulation at the leak point may cause an inflammatory reaction, leading to fibrosis and elimination of the leak (16).

In the current cases, it was not possible to treat the mechanisms causing the failure of lymph drainage, therefore, the selected therapies focused on the peripheral manifestation of the pathological process, treating the lymphorrhea. Dioxide light amplification by the stimulated emission of radiation (CO_2_ laser) was selected, as it is a safe, minimally invasive and repeatable technique, which acts to induce coagulative sclerosis in order to obliterate the subcutaneous and submucosal lymphatic channels, and create a fibrous layer capable of preventing lymphorrhea. Following therapy, a marked reduction in lymphangiectasia associated with increased dermal fibrosis was observed (Fig. 3). This treatment resulted in a decrease in lymphorrhea and pain. The relief of pain may be a consequence of decreased lymphorrhea and damage to the nerve endings near to the treated areas. In the current case, long-term advantages were observed in the two patients, for whom previous lymph drainage and elastic bandaging treatments had been unsuccessful. Quality of life was improved in the patients by reducing the disabling effects of lymphorrhea and its complications; the treatment eliminated the requirement to wear sanitary pads daily, and each patient was able to have sexual intercourse due to the relief from pain. In addition, the second patient experienced no further erysipelas.

Surgical treatment of vulvar lymphorrhea and lymphedema secondary to gynecological cancer treatments remains controversial, and is not currently accepted as standard therapy. The current study utilized laser surgery, a minimally invasive surgical approach to this pathology, which resulted in effective symptomatic treatment. Although this therapy may not be regarded as definitive, as the underlying mechanisms causing the clinical manifestation of lymphedema are not treated, it may provide a valuable long-term treatment strategy. In the present study, the first patient presented with a recurrence of vulvar lymphedema and associated lymphorrhea seven years after the initial laser CO_2_ treatment, and as the treatment is repeatable, further laser CO_2_ surgery could be successfully performed. Therefore, laser CO_2_ surgery has the advantage of being a repeatable technique, which at present has not been reported to have any side effects. The present study indicated that laser CO_2_ surgery is a successful treatment for lymphorrhea, a complication of vulvar lymphedema, however, further studies are required to confirm these findings, using a larger number of patients.

## Figures and Tables

**Figure 1:** Case one: Acanthosis of the overlying squamous epithelium, multiple dilated lymph vessels of varying calibers lined by a single layer of endothelium in the upper dermis, and a lympho-plasmocytic inflammatory infiltrate without giant or atypical cells. Hematoxylin and eosin staining; magnification, ×50.

**Figure 2:** Case two: Marked dilated vessels beneath the epidermis with atrophic changes. Certain vessels contain erythrocytes. Hematoxylin and eosin staining; magnification, ×100.

**Figure 3:** Case two: Isolated lymphangiectasia and normal vessels associated with moderate stromal fibrosis following treatment. Hematoxylin and eosin staining; magnification, ×50.
